The article "An Innovative Decision-Making Approach Based on Correlation Coefficients of Complex Picture Fuzzy Sets and Their Applications in Cluster Analysis" was published in 2022. Journal: Comput Intell Neurosci.

# An Innovative Decision-Making Approach Based on Correlation Coefficients of Complex Picture Fuzzy Sets and Their Applications in Cluster Analysis

**DOI:** 10.1155/2022/7389882

**Published:** 2022-07-08

**Authors:** Jianping Qu, Abdul Nasir, Sami Ullah Khan, Kamsing Nonlaopon, Gauhar Rahman

**Affiliations:** ^1^Information Engineering College, Hebei University of Architecture, Zhangjiakou 075000, China; ^2^Department of Mathematics, Institute of Numerical Sciences, Gomal University, Dera Ismail Khan 29050, Pakistan; ^3^Department of Mathematics, Khon Kaen University, Khon Kaen 40002, Thailand; ^4^Department of Mathematics and Statistics, Hazara University, Mansehra, Pakistan

## Abstract

In modern times, the organizational managements greatly depend on decision-making (DM). DM is considered the management's fundamental function that helps the businesses and organizations to accomplish their targets. Several techniques and processes are proposed for the efficient DM. Sometimes, the situations are unclear and several factors make the process of DM uncertain. Fuzzy set theory has numerous tools to tackle such tentative and uncertain events. The complex picture fuzzy set (CPFS) is a super powerful fuzzy-based structure to cope with the various types of uncertainties. In this article, an innovative DM algorithm is designed which runs for several types of fuzzy information. In addition, a number of new notions are defined which act as the building blocks for the proposed algorithm, such as information energy of a CPFS, correlation between CPFSs, correlation coefficient of CPFSs, matrix of correlation coefficients, and composition of these matrices. Furthermore, some useful results and properties of the novel definitions have been presented. As an illustration, the proposed algorithm is applied to a clustering problem where a company intends to classify its products on the basis of features. Moreover, some experiments are performed for the purpose of comparison. Finally, a comprehensive analysis of the experimental results has been carried out, and the proposed technique is validated.

## 1. Introduction

It is believed that management is actually a process of decision-making (DM). Managing writers claim that an organization accomplishes its long-term and short-term goals through DM. Basically, the act of choosing or selecting an action in a number of actions is known as decision. Thus, DM is the process of opting the most suitable course of action among available choices in order to achieve some target. The direction, planning, organizing, control, and coordination-related matters are solved by DM. Since the entire managerial process is based on decisions, therefore DM plays a vital role in the regulation of a business's performance. Correct decisions reduce diversities, uncertainties, and complexities of the organizational environments. Usually, the following steps are involved in the DM processes to reach deliberate decisions: first, the decision and its nature are identified by gathering enough related information. Then, all the possible alternatives are identified. All of these options are then weighted according to the evidence and expertise. Next, the best choice is being made among the available alternatives based on the information and logical indications. Now, it is the time for action, which means the implementation of the made decision. Finally, the decision is being reviewed and concluding remarks are passed.

The article "An Innovative Decision-Making Approach Based on Correlation Coefficients of Complex Picture Fuzzy Sets and Their Applications in Cluster Analysis" was published in 2022. Journal: Comput Intell Neurosci.

Sighting the complexities and uncertainties in the process of modern DM, mathematicians have worked out different techniques for the purpose. Fuzzy set (FS) theory is a rich field of mathematics that mainly deals with uncertainty, and its major applications are devoted to DM processes. Zadeh [1] conceptualized the FS theory in 1965. It is a set of entities that possess partial memberships. These memberships are actually fuzzy-valued mappings, which means real numbers between 0 and 1 inclusive. Later, in 1986, Atanassov [2] modernized the FS and introduced a structured intuitionistic FS (IFS). These modern sets assign dual functions to their members, known as membership and nonmembership functions. Both of these mappings are fuzzy-valued such that their sum does not exceed 1. In 2013, Cuong and Kreinovich [3] improved the idea of Atanassov by adding a third function to the existing structure. They introduced the world to the notion of picture FS (PFS), where the members of a set possess the membership, abstinence, and nonmembership functions. Each of the mappings is a fuzzy-valued mapping provided that their sum is not greater than 1. Yager [4] used FSs for multiple objective DM, Arfi [5] proposed a linguistic FS approach and applied the concept in political decision making, and Prodanovic and Simonovic [6] compared the FS ranking methods for DM purposes in the implementation of water resources. Based on intuitionistic fuzzy information, Chaira [7] proposed a clustering algorithm with its application to medical images. Dengfeng and Chuntian [8] applied the IFSs in pattern recognition. Lin et al. [9] proposed the multicriterian DM (MCDM) on the basis of IFSs. Singh and Kumar [10] extended the idea of MCDM for PFSs. Si et al. [11] used PFS-based DM in the selection of COVID-19 medications. Van Dinh and Thao [12] applied some measures of PFSs in multiattribute DM (MADM).

In 2003, the structure of FS was adjusted by Ramot et al. [13] such that the membership function was replaced by a complex-valued fuzzy function to propose the edifice of complex FS (CFS). The output values of the membership function in CFS belong to the unit circle in the complex plane. The insertion of imaginary numbers let the framework of CFSs to model dual aspects of a single entity, each represented by real and imaginary numbers. The real part is said to be an amplitude term, while the imaginary part is a phase term. After a decade, in 2012, Alkouri and Salleh [14] came up with the notion of a complex IFS (CIFS). The structures of CIFS and IFS are almost alike. The only difference is the ranges of functions of membership and nonmembership, i.e., they are complex-valued fuzzy mappings. Akram et al. [15] proposed the complex PFS (CPFS) that generalizes all the predescribed fuzzy structures. These are supreme tools to model three properties of an entity with respect to some other variable. Yaqoob et al. [16] used CIFSs in cellular network providers' corporations. Nasir et al. [17–19] applied the CFSs, complex fuzzy relations (CFRs), and their generalizations to cybersecurity and network security. References [20–22] majorly worked on DM methods under the complex fuzzy information.

The article "An Innovative Decision-Making Approach Based on Correlation Coefficients of Complex Picture Fuzzy Sets and Their Applications in Cluster Analysis" was published in 2022. Journal: Comput Intell Neurosci.

In statistical problems, the term correlation coefficient is often used, whose fundamental purpose is to measure the strength of a relationship among entities. Several statisticians and mathematicians have researched the subject of the correlation coefficient. The correlation coefficients are widely used in FS theory. Yang and Lin [23] presented the inclusion and similarity measures for type-2 FS with the application to clustering analysis, Chen et al. [24] also applied the correlation coefficients clustering analysis, Xu et al. [25] gave a clustering algorithm for IFS, Park et al. [26] used the correlation coefficient in the problems of MADM. Garg [27] defined the correlation coefficient for PFS and used it in DM. Some worthwhile research related to decision-making based on uncertainty through fuzzy theory tools includes the remarkable works of Akram et al. [28, 29], who have proposed different clustering algorithms. Ganie et al. [30] defined the correlation coefficients of PFS and applied them in medical diagnosis.

Espying the development of practical applications of correlation coefficients in the theory of FSs, this research is ardent to propose some innovative DM techniques based on correlation coefficients. To this end, the information energy of a CPFS, the correlation between two CPFSs, and the correlation coefficient of CPFSs are defined, which act as the building blocks for the proposed DM algorithm. Furthermore, the matrix of correlation coefficients for more than one CPFS is established, which is followed by the definitions of the equivalence matrix and the composition of the matrix of correlation coefficients. In addition, the *α*-cutting classification rules are described. Many interesting properties and worthwhile results have been proposed for the proposed definitions. Moreover, the clustering algorithm based on correlation coefficients of CPFSs is designed. As an illustration, the proposed algorithm is applied to solve the problem of classifying the set of laptops on the basis of specifications and features. Several experiments are carried out to validate the working and supremacy of the proposed algorithm as compared to the rest of the available techniques in the literature. Finally, the experimental section ends with the remarks stating the advantages of proposed method and the limitations of existing methods. The proposed methods can be used in a wide range of problems, and they are capable of dealing with a large variety of data. The practicality of the given methods includes their applications to pattern recognition as Yang and Yang [31], for example, the pattern recognition in the construction of buildings and the materials [32] and medical diagnosis [30]. Moreover, it could be successfully used to categorize the masks' types on the basis of their characteristics, i.e., some are used for dust prevention, others are clinical masks, COVID-19 preventive masks, and masks made of clothes. In the future, the proposed structures and ideas could be extended to other generalizations of fuzzy theory, especially the spherical fuzzy structures that permit the decision-makers to work in a greater domain as compared to the other frameworks. Henceforth, it would be worthwhile to cover those regions with the novel techniques of this paper. The introduction section is followed by the preliminaries section, which comprises some basic definitions such as FS, CFS, IFS, CIFS, PFS, CPFS, and correlation coefficient of IFSs. The third section proposes the correlation coefficients for the CPFSs along with some results and properties. In Section 4, the clustering algorithm based on proposed concepts is designed. Section 5 is devoted to the application of the designed algorithm for CPFSs. In Section 6, the experimental comparisons are carried out, which states the advantages of proposed structures and disadvantages of other methods. Finally, Section 7 concludes this research.

The article "An Innovative Decision-Making Approach Based on Correlation Coefficients of Complex Picture Fuzzy Sets and Their Applications in Cluster Analysis" was published in 2022. Journal: Comput Intell Neurosci.

## 2. Preliminaries

In this section, the definitions of some fundamental concepts are presented, which will be used for the further research. First, we define the fuzzy set (FS), which was presented by Zadeh [1].

**Definition 1 (see [1]).**

Let *R* denote the referential or universal set. Then an FS denoted by *Z* is of the form *Z*={*z*, *ξ*(*z*) : *z* ∈ *R*}, where the entity *ξ*(*z*) is called the membership function, which assigns each of the elements of *R* (i.e., *z* ∈ *R*) a fuzzy number (FN) *N*, i.e., *N* ∈ [0,1].

Now, the intuitionistic fuzzy set (IFS) is defined, which was introduced by Atanassov [2].

**Definition 2 (see [2]).**

Let *R* denote the referential set. Then an IFS denoted by *Z* is of the form *Z*={*z*, *ξ*(*z*), *η*(*z*) : *z* ∈ *R*}, where the entities *ξ*(*z*) and *η*(*z*) are called the membership and nonmembership functions, respectively, which assign each of the elements of *R* (i.e., *z* ∈ *R*) FNs *N*_1_ and *N*_2_, respectively, given that their sum is also a FN, i.e., *N*_1_, *N*_2_ ∈ [0,1]∋*N*_1_+*N*_2_ ∈ [0,1].

Now, the definition of picture fuzzy set (PFS) was given by Cuong et al. [3] as follows.

**Definition 3 (see [3]).**

Let *R* denote the referential set. Then a PFS denoted by *Z* is of the form *Z*={*z*, *ξ*(*z*), *α*(*z*), *η*(*z*) : *z* ∈ *R*}, where the entities *ξ*(*z*), *α*(*z*), and *η*(*z*) are called the membership, abstinence, and nonmembership functions, respectively, which assign each of the elements of *R* (i.e., *z* ∈ *R*) FNs *N*_1_, *N*_2_, and *N*_3_, respectively, given that their sum is also a FN, i.e., *N*_1_, *N*_2_, *N*_3_ ∈ [0,1]∋*N*_1_+*N*_2_+*N*_3_ ∈ [0,1].

Ramot et al. [13] defined the complex fuzzy set (CFS) as follows.

**Definition 4 (see [13]).**

Let *R* denote the referential set. Then a CFS denoted by *Z* is of the form *Z*={*z*, *ξ*(*z*)*e*^*ρ*(*z*)2*πi*^ : *z* ∈ *R*}, where the entity *ξ*(*z*) and *ρ*(*z*) are called the amplitude and phase terms of membership function, respectively, which assign each of the elements of *R* (i.e., *z* ∈ *R*) a fuzzy number (FN) *N*, i.e., *N* ∈ [0,1].

Later, Alkouri and Salleh [14] came up with the notion of a complex IFS (CIFS).

**Definition 5 (see [14]).**

Let *R* denote the referential set. Then a CIFS denoted by *Z* is of the form *Z*={*z*, *ξ*(*z*)*e*^*ρ*_*ξ*_(*z*)2*πi*^, *η*(*z*)*e*^*ρ*_*η*_(*z*)2*πi*^ : *z* ∈ *R*}, where the entities *ξ*(*z*) and *η*(*z*) are called the amplitude terms of membership and nonmembership functions, respectively, which assign each of the elements of *R* (i.e., *z* ∈ *R*) FNs *N*_1_ and *N*_2_, respectively, given that their sum is also a FN, i.e., *N*_1_, *N*_2_ ∈ [0,1]∋*N*_1_+*N*_2_ ∈ [0,1]. Likewise, the entities *ρ*_*ξ*_(*z*) and *ρ*_*η*_(*z*) are called the phase terms of membership and nonmembership functions, respectively, which also assign each of the elements of *R* (i.e., *z* ∈ *R*) FNs *N*_3_ and *N*_4_, respectively, given that their sum is also a FN, i.e., *N*_3_, *N*_4_ ∈ [0,1]∋*N*_3_+*N*_4_ ∈ [0,1].

The article "An Innovative Decision-Making Approach Based on Correlation Coefficients of Complex Picture Fuzzy Sets and Their Applications in Cluster Analysis" was published in 2022. Journal: Comput Intell Neurosci.

Akram et al. [15] proposed the complex PFS (CPFS) that generalizes all the predescribed fuzzy structures.

**Definition 6 (see [15]).**

Let *R* denote the referential set. Then a CPFS denoted by *Z* is of the form *Z*={*z*, *ξ*(*z*)*e*^*ρ*_*ξ*_(*z*)2*πi*^, *α*(*z*)*e*^*ρ*_*α*_(*z*)2*πi*^, *η*(*z*)*e*^*ρ*_*η*_(*z*)2*πi*^ : *z* ∈ *R*}, where the entities *ξ*(*z*), *α*(*z*) and *η*(*z*) are called the amplitude terms of membership, abstinence, and nonmembership functions, respectively, which assign each of the elements of *R* (i.e., *z* ∈ *R*) FNs *N*_1_, *N*_2_, and *N*_3_, respectively, given that their sum is also a FN, i.e., *N*_1_, *N*_2_, *N*_3_ ∈ [0,1]∋*N*_1_+*N*_2_+*N*_3_ ∈ [0,1]. Likewise, the entities *ρ*_*ξ*_(*z*), *ρ*_*α*_(*z*), and *ρ*_*η*_(*z*) are called the phase terms of membership, abstinence, and nonmembership functions, respectively, which also assign each of the elements of *R* (i.e., *z* ∈ *R*) FNs *N*_4_, *N*_5_, and *N*_6_, respectively, given that their sum is also a FN, i.e., *N*_4_, *N*_5_, *N*_6_ ∈ [0,1]∋*N*_4_+*N*_5_+*N*_6_ ∈ [0,1].

Figure 1 depicts a summary of generalizations of CPFSs in the light of above definitions.

Now, the information energy (IE) of an IFS, correlation of IFSs, and correlation coefficient of IFSs are defined in the following definitions.

**Definition 7 (see [25]).**

Let *Z*={*z*, *ξ*(*z*), *η*(*z*) : *z* ∈ *R*} be an IFS on a referential set *R*, then its information energy (IE) denoted by *ℰ* is calculated by

(1) $$\begin{array}{c} E\left(Z\right)=\overset{n}{\underset{k=1}{\sum }}\left[{\left(\xi \left(z_{k}\right)\right)}^{2}+{\left(\eta \left(z_{k}\right)\right)}^{2}\right]. \end{array}$$

**Definition 8 (see [25]).**

Let *Y*={*y*, *ξ*(*y*), *η*(*y*) : *y* ∈ *R*} and *Z*={*z*, *ξ*(*z*), *η*(*z*) : *z* ∈ *R*} be any IFSs on a referential set *R*, then their correlation denoted by Δ is calculated by

(2) $$\begin{array}{c} \Delta \left(Y,Z\right)=\overset{n}{\underset{k=1}{\sum }}\left[\xi \left(y_{k}\right)\times \xi \left(z_{k}\right)+\eta \left(y_{k}\right)\times \eta \left(z_{k}\right)\right]. \end{array}$$

**Definition 9 (see [25]).**

Let *Y*={*y*, *ξ*(*y*), *η*(*y*) : *y* ∈ *R*} and *Z*={*z*, *ξ*(*z*), *η*(*z*) : *z* ∈ *R*} be any IFSs on a referential set *R*, then their correlation coefficient denoted by ∁ is calculated by formula (3) or alternatively formula (4):

(3) $$\begin{array}{c} ∁\left(Y,Z\right)=\frac{\Delta \left(Y,Z\right)}{\sqrt{\left[E\left(Y\right)\times E\left(Z\right)\right]}}, \end{array}$$

(4) $$\begin{array}{c} =\frac{\sum_{k=1}^{n}\left[\xi \left(y_{k}\right)\times \xi \left(z_{k}\right)+\eta \left(y_{k}\right)\times \eta \left(z_{k}\right)\right]}{\sqrt{\sum_{k=1}^{n}\left[{\left(\xi \left(y_{k}\right)\right)}^{2}+{\left(\eta \left(y_{k}\right)\right)}^{2}\right]\times \sum_{k=1}^{n}\left[{\left(\xi \left(z_{k}\right)\right)}^{2}+{\left(\eta \left(z_{k}\right)\right)}^{2}\right]}}. \end{array}$$

The article "An Innovative Decision-Making Approach Based on Correlation Coefficients of Complex Picture Fuzzy Sets and Their Applications in Cluster Analysis" was published in 2022. Journal: Comput Intell Neurosci.

## 3. Correlation Coefficient for Complex Picture Fuzzy Sets

This section is intended to give the formulae to calculate the IE, correlation, and correlation coefficients for CPFSs.

**Definition 10 .**

Let *Z*={*z*, *ξ*(*z*)*e*^*ρ*_*ξ*_(*z*)2*πi*^, *α*(*z*)*e*^*ρ*_*α*_(*z*)2*πi*^, *η*(*z*)*e*^*ρ*_*η*_(*z*)2*πi*^ : *z* ∈ *R*} be a CPFS on a referential set *R*, then its information energy (IE) denoted by *ℰ* is calculated by

(5) $$\begin{array}{c} E\left(Z\right)=\overset{n}{\underset{k=1}{\sum }}\left[\left({\left(\xi \left(z_{k}\right)\right)}^{2}+{\left(\alpha \left(z_{k}\right)\right)}^{2}+{\left(\eta \left(z_{k}\right)\right)}^{2}\right)+\left({\left(\rho_{\xi }\left(z_{k}\right)\right)}^{2}+{\left(\rho_{\alpha }\left(z_{k}\right)\right)}^{2}+{\left(\rho_{\eta }\left(z_{k}\right)\right)}^{2}\right)\right]. \end{array}$$

**Definition 11 .**

Let *Y*={*y*, *ξ*(*y*)*e*^*ρ*_*ξ*_(*y*)2*πi*^, *α*(*y*)*e*^*ρ*_*α*_(*y*)2*πi*^, *η*(*y*)*e*^*ρ*_*η*_(*y*)2*πi*^ : *y* ∈ *R*} and *Z*={*z*, *ξ*(*z*)*e*^*ρ*_*ξ*_(*z*)2*πi*^, *α*(*z*)*e*^*ρ*_*α*_(*z*)2*πi*^, *η*(*z*)*e*^*ρ*_*η*_(*z*)2*πi*^ : *z* ∈ *R*} be any CPFSs on a referential set *R*, then their correlation denoted by Δ is calculated by

(6) $$\begin{array}{c} \Delta \left(Y,Z\right)=\overset{n}{\underset{k=1}{\sum }}\left[\begin{array}{c} \left(\xi \left(y_{k}\right)\times \xi \left(z_{k}\right)+\alpha \left(y_{k}\right)\times \alpha \left(z_{k}\right)+\eta \left(y_{k}\right)\times \eta \left(z_{k}\right)\right)+\\ \left(\rho_{\xi }\left(y_{k}\right)\times \rho_{\xi }\left(z_{k}\right)+\rho_{\alpha }\left(y_{k}\right)\times \rho_{\alpha }\left(z_{k}\right)+\rho_{\eta }\left(y_{k}\right)\times \rho_{\eta }\left(z_{k}\right)\right) \end{array}\right]. \end{array}$$

**Definition 12 .**

Let *Y*={*y*, *ξ*(*y*)*e*^*ρ*_*ξ*_(*y*)2*πi*^, *α*(*y*)*e*^*ρ*_*α*_(*y*)2*πi*^, *η*(*y*)*e*^*ρ*_*η*_(*y*)2*πi*^ : *y* ∈ *R*} and *Z*={*z*, *ξ*(*z*)*e*^*ρ*_*ξ*_(*z*)2*πi*^, *α*(*z*)*e*^*ρ*_*α*_(*z*)2*πi*^, *η*(*z*)*e*^*ρ*_*η*_(*z*)2*πi*^ : *z* ∈ *R*} be any CPFSs on a referential set *R*, then their correlation coefficient denoted by ∁ is calculated by formula (7) or alternatively formula (8):

(7) $$\begin{array}{c} ∁\left(Y,Z\right)=\frac{\Delta \left(Y,Z\right)}{\sqrt{\left[E\left(Y\right)\times E\left(Z\right)\right]}}, \end{array}$$

(8) $$\begin{array}{c} =\frac{\sum_{k=1}^{n}\left[\begin{array}{c} \left(\xi \left(y_{k}\right)\times \xi \left(z_{k}\right)+\alpha \left(y_{k}\right)\times \alpha \left(z_{k}\right)+\eta \left(y_{k}\right)\times \eta \left(z_{k}\right)\right)+\\ \left(\rho_{\xi }\left(y_{k}\right)\times \rho_{\xi }\left(z_{k}\right)+\rho_{\alpha }\left(y_{k}\right)\times \rho_{\alpha }\left(z_{k}\right)+\rho_{\eta }\left(y_{k}\right)\times \rho_{\eta }\left(z_{k}\right)\right) \end{array}\right]}{\sqrt{\left[\begin{array}{c} \sum_{k=1}^{n}\left[\left({\left(\xi \left(y_{k}\right)\right)}^{2}+{\left(\alpha \left(y_{k}\right)\right)}^{2}+{\left(\eta \left(y_{k}\right)\right)}^{2}\right)+\left({\left(\rho_{\xi }\left(y_{k}\right)\right)}^{2}+{\left(\rho_{\alpha }\left(y_{k}\right)\right)}^{2}+{\left(\rho_{\eta }\left(y_{k}\right)\right)}^{2}\right)\right]\times \\ \sum_{k=1}^{n}\left[\left({\left(\xi \left(z_{k}\right)\right)}^{2}+{\left(\alpha \left(z_{k}\right)\right)}^{2}+{\left(\eta \left(z_{k}\right)\right)}^{2}\right)+\left({\left(\rho_{\xi }\left(z_{k}\right)\right)}^{2}+{\left(\rho_{\alpha }\left(z_{k}\right)\right)}^{2}+{\left(\rho_{\eta }\left(z_{k}\right)\right)}^{2}\right)\right] \end{array}\right]}}. \end{array}$$

**Theorem 1 .**

The article "An Innovative Decision-Making Approach Based on Correlation Coefficients of Complex Picture Fuzzy Sets and Their Applications in Cluster Analysis" was published in 2022. Journal: Comput Intell Neurosci.

Let ∁(*Y*, *Z*) be the correlation coefficient for CPFSs *Y* and *Z*. Then,

- It is symmetric, i.e., ∁(*Y*, *Z*)=∁(*Z*, *Y*)
- It is an FN, i.e., 0 ≤ ∁(*Y*, *Z*) ≤ 1
- ∁(*Y*, *Z*)=1⇔*Y*=*Z*.

**Proof**

(i) The substitution of values on both sides and simplification proves the first claim.
(ii) As ∁(*Y*, *Z*) is calculated by using the values of membership, abstinence, and nonmembership functions of CPFSs *Y* and *Z*, therefore ∁(*Y*, *Z*) ≥ 0. For the other part of inequality, i.e., ∁(*Y*, *Z*) ≤ 1, consider the Δ(*Y*, *Z*).
  (9) $$\begin{array}{c} \Delta \left(Y,Z\right)=\overset{n}{\underset{k=1}{\sum }}\left[\begin{array}{c} \left(\xi \left(y_{k}\right)\times \xi \left(z_{k}\right)+\alpha \left(y_{k}\right)\times \alpha \left(z_{k}\right)+\eta \left(y_{k}\right)\times \eta \left(z_{k}\right)\right)+\\ \left(\rho_{\xi }\left(y_{k}\right)\times \rho_{\xi }\left(z_{k}\right)+\rho_{\alpha }\left(y_{k}\right)\times \rho_{\alpha }\left(z_{k}\right)+\rho_{\eta }\left(y_{k}\right)\times \rho_{\eta }\left(z_{k}\right)\right) \end{array}\right]\\ =\left[\begin{array}{c} \left(\xi \left(y_{1}\right)\times \xi \left(z_{1}\right)+\alpha \left(y_{1}\right)\times \alpha \left(z_{1}\right)+\eta \left(y_{1}\right)\times \eta \left(z_{1}\right)\right)+\\ \left(\rho_{\xi }\left(y_{1}\right)\times \rho_{\xi }\left(z_{1}\right)+\rho_{\alpha }\left(y_{1}\right)\times \rho_{\alpha }\left(z_{1}\right)+\rho_{\eta }\left(y_{1}\right)\times \rho_{\eta }\left(z_{1}\right)\right) \end{array}\right]\\ +\left[\begin{array}{c} \left(\xi \left(y_{2}\right)\times \xi \left(z_{2}\right)+\alpha \left(y_{2}\right)\times \alpha \left(z_{2}\right)+\eta \left(y_{2}\right)\times \eta \left(z_{2}\right)\right)+\\ \left(\rho_{\xi }\left(y_{2}\right)\times \rho_{\xi }\left(z_{2}\right)+\rho_{\alpha }\left(y_{2}\right)\times \rho_{\alpha }\left(z_{2}\right)+\rho_{\eta }\left(y_{2}\right)\times \rho_{\eta }\left(z_{2}\right)\right) \end{array}\right]+\cdots \\ +\left[\begin{array}{c} \left(\xi \left(y_{n}\right)\times \xi \left(z_{n}\right)+\alpha \left(y_{n}\right)\times \alpha \left(z_{n}\right)+\eta \left(y_{n}\right)\times \eta \left(z_{n}\right)\right)+\\ \left(\rho_{\xi }\left(y_{n}\right)\times \rho_{\xi }\left(z_{n}\right)+\rho_{\alpha }\left(y_{n}\right)\times \rho_{\alpha }\left(z_{n}\right)+\rho_{\eta }\left(y_{n}\right)\times \rho_{\eta }\left(z_{n}\right)\right) \end{array}\right]. \end{array}$$
According to the statement of Cauchy Schwarz; for (*y*_1_, *y*_2_,…, *y*_*n*_), (*z*_1_, *z*_2_,…, *z*_*n*_) ∈ ℝ^*n*^, where ℝ is set of real numbers, imply
  (10) $$\begin{array}{c} \sqrt{\left(y_{1}z_{1}+y_{2}z_{2}+y_{3}z_{3}+\ldots +y_{n}z_{n}\right)}\leq \left(y_{1}^{2}+y_{2}^{2}+\ldots +y_{n}^{2}\right)\times \left(z_{1}^{2}+z_{2}^{2}+\ldots +z_{n}^{2}\right). \end{array}$$
Thus, by applying the Cauchy Schwarz inequality to above stated equation for Δ(*Y*, *Z*) implies
  (11) $$\begin{array}{c} {\left(\Delta \left(Y,Z\right)\right)}^{2}\leq \left[\begin{array}{c} \left(\begin{array}{c} {\left(\left(\xi \left(y_{1}\right)\right)\right)}^{2}+{\left(\alpha \left(y_{1}\right)\right)}^{2}+{\left(\eta \left(y_{1}\right)\right)}^{2}+\left({\left(\rho \xi \left(y_{1}\right)\right)}^{2}+{\left(\rho \alpha \left(y_{1}\right)\right)}^{2}+{\left(\rho \eta \left(y_{1}\right)\right)}^{2}\right)+\\ \left({\left(\xi \left(y_{2}\right)\right)}^{2}+{\left(\alpha \left(y_{2}\right)\right)}^{2}+{\left(\eta \left(y_{2}\right)\right)}^{2}\right)+\left({\left(\rho \xi \left(y_{2}\right)\right)}^{2}+{\left(\rho \alpha \left(y_{2}\right)\right)}^{2}+{\left(\rho \eta \left(y_{2}\right)\right)}^{2}\right)+\ldots +\\ {\left(\left(\xi \left(y_{n}\right)\right)\right)}^{2}+{\left(\alpha \left(y_{n}\right)\right)}^{2}+{\left(\eta \left(y_{n}\right)\right)}^{2}+\left({\left(\rho \xi \left(y_{n}\right)\right)}^{2}+{\left(\rho \alpha \left(y_{n}\right)\right)}^{2}+{\left(\rho \eta \left(y_{n}\right)\right)}^{2}\right) \end{array}\right)\times \\ \left(\begin{array}{c} {\left(\left(\xi \left(z_{1}\right)\right)\right)}^{2}+{\left(\alpha \left(z_{1}\right)\right)}^{2}+{\left(\eta \left(z_{1}\right)\right)}^{2}+\left({\left(\rho \xi \left(z_{1}\right)\right)}^{2}+{\left(\rho \alpha \left(z_{1}\right)\right)}^{2}+{\left(\rho \eta \left(z_{1}\right)\right)}^{2}\right)+\\ \left({\left(\xi \left(z_{2}\right)\right)}^{2}+{\left(\alpha \left(z_{2}\right)\right)}^{2}+{\left(\eta \left(z_{2}\right)\right)}^{2}\right)+\left({\left(\rho \xi \left(z_{2}\right)\right)}^{2}+{\left(\rho \alpha \left(z_{2}\right)\right)}^{2}+{\left(\rho \eta \left(z_{2}\right)\right)}^{2}\right)+\ldots +\\ {\left(\left(\xi \left(z_{n}\right)\right)\right)}^{2}+{\left(\alpha \left(z_{n}\right)\right)}^{2}+{\left(\eta \left(z_{n}\right)\right)}^{2}+\left({\left(\rho \xi \left(z_{n}\right)\right)}^{2}+{\left(\rho \alpha \left(z_{n}\right)\right)}^{2}+{\left(\rho \eta \left(z_{n}\right)\right)}^{2}\right) \end{array}\right) \end{array}\right]\\ =\left[\begin{array}{c} \overset{n}{\underset{k=1}{\sum }}\left(\left({\left(\xi \left(y_{k}\right)\right)}^{2}+{\left(\alpha \left(y_{k}\right)\right)}^{2}+{\left(\eta \left(y_{k}\right)\right)}^{2}\right)+\left({\left(\rho_{\xi }\left(y_{k}\right)\right)}^{2}+{\left(\rho_{\alpha }\left(y_{k}\right)\right)}^{2}+{\left(\rho_{\eta }\left(y_{k}\right)\right)}^{2}\right)\right)\times \\ \overset{n}{\underset{k=1}{\sum }}\left(\left({\left(\xi \left(z_{k}\right)\right)}^{2}+{\left(\alpha \left(z_{k}\right)\right)}^{2}+{\left(\eta \left(z_{k}\right)\right)}^{2}\right)+\left({\left(\rho_{\xi }\left(z_{k}\right)\right)}^{2}+{\left(\rho_{\alpha }\left(z_{k}\right)\right)}^{2}+{\left(\rho_{\eta }\left(z_{k}\right)\right)}^{2}\right)\right) \end{array}\right]\\ =E\left(Y\right)\times E\left(Z\right) \end{array}$$
Thus, ${\left(\Delta \left(Y,Z\right)\right)}^{2}\leq ℰ\left(Y\right)\times ℰ\left(Z\right)\Rightarrow \left(\Delta \left(Y,Z\right)\right)\leq \sqrt{ℰ\left(Y\right)\times ℰ\left(Z\right)}\Rightarrow \left(\left(\Delta \left(Y,Z\right)\right)/\sqrt{ℰ\left(Y\right)\times ℰ\left(Z\right)}\right)\leq 1$.
Hence, 0 ≤ ∁(*Y*, *Z*) ≤ 1.
(iii) For *Y*=*Z*⇔*ξ*(*y*_*k*_)=*ξ*(*z*_*k*_), *α*(*y*_*k*_)=*α*(*z*_*k*_), *η*(*y*_*k*_)=*η*(*z*_*k*_), *ρ*_*ξ*_(*y*_*k*_)=*ρ*_*ξ*_(*z*_*k*_), *ρ*_*α*_(*y*_*k*_)=*ρ*_*α*_(*z*_*k*_) and *ρ*_*η*_(*y*_*k*_)=*ρ*_*η*_(*z*_*k*_) where *y*_*k*_, *z*_*k*_ ∈ *R*. Thus, ∁(*Y*, *Z*)=1

**Example 1 .**

The article "An Innovative Decision-Making Approach Based on Correlation Coefficients of Complex Picture Fuzzy Sets and Their Applications in Cluster Analysis" was published in 2022. Journal: Comput Intell Neurosci.

Suppose *Y* and *Z* are two CPFS on *R*={*y*_1_, *y*_2_, *y*_3_, *z*_1_, *z*_2_, *z*_3_} stated as

(12) $$\begin{array}{c} Y=\left\{\begin{array}{c} \left(y_{1},0.3e^{2\pi i\left(0.1\right)},0.5e^{2\pi i\left(0.4\right)},0.1e^{2\pi i\left(0.3\right)}\right),\\ \left(y_{2},0.4e^{2\pi i\left(0.3\right)},0.2e^{2\pi i\left(0.3\right)},0.2e^{2\pi i\left(0.3\right)}\right),\\ \left(y_{3},0.2e^{2\pi i\left(0.4\right)},0.1e^{2\pi i\left(0.4\right)},0.7e^{2\pi i\left(0.1\right)}\right) \end{array}\right\},\\ Z=\left\{\begin{array}{c} \left(z_{1},0.2e^{2\pi i\left(0.6\right)},0.4e^{2\pi i\left(0.1\right)},0.3e^{2\pi i\left(0.2\right)}\right),\\ \left(z_{2},0.3e^{2\pi i\left(0.4\right)},0.3e^{2\pi i\left(0.3\right)},0.4e^{2\pi i\left(0.1\right)}\right),\\ \left(z_{3},0.5e^{2\pi i\left(0.1\right)},0.4e^{2\pi i\left(0.5\right)},0.1e^{2\pi i\left(0.3\right)}\right) \end{array}\right\}. \end{array}$$

Then by using formula (5), the IE of *Y* and *Z* are calculated as

(13) $$\begin{array}{c} E\left(Y\right)=1.99, \end{array}$$

(14) $$\begin{array}{c} E\left(Z\right)=2.07. \end{array}$$

Also, by using formula (6), the correlation of *Y* and *Z* is calculated as

(15) $$\begin{array}{c} \Delta \left(Y,Z\right)=1.43. \end{array}$$

Moreover, by using formula (8), the correlation coefficient of Y and *Z* is calculated as

(16) $$\begin{array}{c} ∁\left(Y,Z\right)=0.704. \end{array}$$

There is an alternative way of calculating the correlation coefficient for CPFSs.

**Definition 13 .**

Let *Y*={*y*, *ξ*(*y*)*e*^*ρ*_*ξ*_(*y*)2*πi*^, *α*(*y*)*e*^*ρ*_*α*_(*y*)2*πi*^, *η*(*y*)*e*^*ρ*_*η*_(*y*)2*πi*^ : *y* ∈ *R*} and *Z*={*z*, *ξ*(*z*)*e*^*ρ*_*ξ*_(*z*)2*πi*^, *α*(*z*)*e*^*ρ*_*α*_(*z*)2*πi*^, *η*(*z*)*e*^*ρ*_*η*_(*z*)2*πi*^ : *z* ∈ *R*} be any CPFSs on a referential set *R*, then their correlation coefficient denoted by ∁' is also calculated by formula (18) or alternatively formula (19):

(17) $$\begin{array}{c} {∁}^{\prime }\left(Y,Z\right)=\frac{\Delta \left(Y,Z\right)}{\max\left\{\Delta \left(Y,Y\right),\Delta \left(Z,Z\right)\right\}}, \end{array}$$

(18) $$\begin{array}{c} =\frac{\sum_{k=1}^{n}\left[\begin{array}{c} \left(\xi \left(y_{k}\right)\times \xi \left(z_{k}\right)+\alpha \left(y_{k}\right)\times \alpha \left(z_{k}\right)+\eta \left(y_{k}\right)\times \eta \left(z_{k}\right)\right)+\\ \left(\rho_{\xi }\left(y_{k}\right)\times \rho_{\xi }\left(z_{k}\right)+\rho_{\alpha }\left(y_{k}\right)\times \rho_{\alpha }\left(z_{k}\right)+\rho_{\eta }\left(y_{k}\right)\times \rho_{\eta }\left(z_{k}\right)\right) \end{array}\right]}{\max\left\{\begin{array}{c} \sum_{k=1}^{n}\left[\left({\left(\xi \left(y_{k}\right)\right)}^{2}+{\left(\alpha \left(y_{k}\right)\right)}^{2}+{\left(\eta \left(y_{k}\right)\right)}^{2}\right)+\left({\left(\rho_{\xi }\left(y_{k}\right)\right)}^{2}+{\left(\rho_{\alpha }\left(y_{k}\right)\right)}^{2}+{\left(\rho_{\eta }\left(y_{k}\right)\right)}^{2}\right)\right],\\ \sum_{k=1}^{n}\left[\left({\left(\xi \left(z_{k}\right)\right)}^{2}+{\left(\alpha \left(z_{k}\right)\right)}^{2}+{\left(\eta \left(z_{k}\right)\right)}^{2}\right)+\left({\left(\rho_{\xi }\left(z_{k}\right)\right)}^{2}+{\left(\rho_{\alpha }\left(z_{k}\right)\right)}^{2}+{\left(\rho_{\eta }\left(z_{k}\right)\right)}^{2}\right)\right] \end{array}\right\}}. \end{array}$$

Now, Theorem 1 is proved using the alternative definition of correlation coefficient as follows.

The article "An Innovative Decision-Making Approach Based on Correlation Coefficients of Complex Picture Fuzzy Sets and Their Applications in Cluster Analysis" was published in 2022. Journal: Comput Intell Neurosci.

**Theorem 2 .**

Let *∁*′(*Y*, *Z*) be the correlation coefficient for CPFSs *Y* and *Z*. Then,

- It is symmetric, i.e., *∁*′(*Y*, *Z*)=*∁*′(*Z*, *Y*)
- It is an FN, i.e., 0 ≤ *∁*′(*Y*, *Z*) ≤ 1
- *∁*′(*Y*, *Z*)=1⇔*Y*=*Z*.

**Proof**

(i) The substitution of values on both sides and simplification proves the first claim.
(ii) Obviously *∁*′(*Y*, *Z*) ≥ 0. By using Theorem 1, the following is implied:
  (19) $$\begin{array}{c} \Delta \left(Y,Z\right)\leq \sqrt{\Delta \left(Y,Y\right)\times \Delta \left(Z,Z\right)}. \end{array}$$
Therefore,
  (20) $$\begin{array}{c} \Delta \left(Y,Z\right)\leq \max\left\{\Delta \left(Y,Y\right),\Delta \left(Z,Z\right)\right\}. \end{array}$$
Hence, *∁*′(*Y*, *Z*) ≤ 1.
(iii) The proof is straight forward.

As far as the applications and practicality is concerned, the weight value of an expert's opinion acts as a crucial part in problems concerning multiattribute decision-making (MADM). Each of the attributes carries a particular weight value. Henceforth, it is essential to develop some weighted correlation coefficients. A vector of weight values is defined and denoted by *Ω*=(*ω*_1_, *ω*_2_,…, *ω*_*n*_)∋*ω*_*k*_ ≥ 0 and ∑_*k*=1_^*n*^*ω*_*k*_=1, where *k* ∈ {1,2,3,…*n*}.

**Definition 14 .**

Let *Y*={*y*, *ξ*(*y*)*e*^*ρ*_*ξ*_(*y*)2*πi*^, *α*(*y*)*e*^*ρ*_*α*_(*y*)2*πi*^, *η*(*y*)*e*^*ρ*_*η*_(*y*)2*πi*^ : *y* ∈ *R*} and *Z*={*z*, *ξ*(*z*)*e*^*ρ*_*ξ*_(*z*)2*πi*^, *α*(*z*)*e*^*ρ*_*α*_(*z*)2*πi*^, *η*(*z*)*e*^*ρ*_*η*_(*z*)2*πi*^ : *z* ∈ *R*} be any CPFSs on a referential set *R*, then their weighted correlation coefficient denoted by ∁_*Ω*_ is calculated by

(21) $$\begin{array}{c} {∁}_{\Omega }=\frac{\sum_{k=1}^{n}\left(\omega_{k}\right)\left[\begin{array}{c} \left(\xi \left(y_{k}\right)\times \xi \left(z_{k}\right)+\alpha \left(y_{k}\right)\times \alpha \left(z_{k}\right)+\eta \left(y_{k}\right)\times \eta \left(z_{k}\right)\right)+\\ \left(\rho_{\xi }\left(y_{k}\right)\times \rho_{\xi }\left(z_{k}\right)+\rho_{\alpha }\left(y_{k}\right)\times \rho_{\alpha }\left(z_{k}\right)+\rho_{\eta }\left(y_{k}\right)\times \rho_{\eta }\left(z_{k}\right)\right) \end{array}\right]}{\sqrt{\left[\begin{array}{c} \sum_{k=1}^{n}\left(\omega_{k}\right)\left[\left({\left(\xi \left(y_{k}\right)\right)}^{2}+{\left(\alpha \left(y_{k}\right)\right)}^{2}+{\left(\eta \left(y_{k}\right)\right)}^{2}\right)+\left({\left(\rho_{\xi }\left(y_{k}\right)\right)}^{2}+{\left(\rho_{\alpha }\left(y_{k}\right)\right)}^{2}+{\left(\rho_{\eta }\left(y_{k}\right)\right)}^{2}\right)\right]\times \\ \sum_{k=1}^{n}\left(\omega_{k}\right)\left[\left({\left(\xi \left(z_{k}\right)\right)}^{2}+{\left(\alpha \left(z_{k}\right)\right)}^{2}+{\left(\eta \left(z_{k}\right)\right)}^{2}\right)+\left({\left(\rho_{\xi }\left(z_{k}\right)\right)}^{2}+{\left(\rho_{\alpha }\left(z_{k}\right)\right)}^{2}+{\left(\rho_{\eta }\left(z_{k}\right)\right)}^{2}\right)\right] \end{array}\right]}}. \end{array}$$

**Definition 15 .**

The article "An Innovative Decision-Making Approach Based on Correlation Coefficients of Complex Picture Fuzzy Sets and Their Applications in Cluster Analysis" was published in 2022. Journal: Comput Intell Neurosci.

Let *Y*={*y*, *ξ*(*y*)*e*^*ρ*_*ξ*_(*y*)2*πi*^, *α*(*y*)*e*^*ρ*_*α*_(*y*)2*πi*^, *η*(*y*)*e*^*ρ*_*η*_(*y*)2*πi*^ : *y* ∈ *R*} and *Z*={*z*, *ξ*(*z*)*e*^*ρ*_*ξ*_(*z*)2*πi*^, *α*(*z*)*e*^*ρ*_*α*_(*z*)2*πi*^, *η*(*z*)*e*^*ρ*_*η*_(*z*)2*πi*^ : *z* ∈ *R*} be any CPFSs on a referential set *R*, then their weighted correlation coefficient denoted by ∁_*Ω*_′ is also calculated by

(22) $$\begin{array}{c} {∁}_{\Omega }^{\prime }=\frac{\sum_{k=1}^{n}\left(\omega_{k}\right)\left[\begin{array}{c} \left(\xi \left(y_{k}\right)\times \xi \left(z_{k}\right)+\alpha \left(y_{k}\right)\times \alpha \left(z_{k}\right)+\eta \left(y_{k}\right)\times \eta \left(z_{k}\right)\right)+\\ \left(\rho_{\xi }\left(y_{k}\right)\times \rho_{\xi }\left(z_{k}\right)+\rho_{\alpha }\left(y_{k}\right)\times \rho_{\alpha }\left(z_{k}\right)+\rho_{\eta }\left(y_{k}\right)\times \rho_{\eta }\left(z_{k}\right)\right) \end{array}\right]}{\max\left\{\begin{array}{c} \sum_{k=1}^{n}\left(\omega_{k}\right)\left[\left({\left(\xi \left(y_{k}\right)\right)}^{2}+{\left(\alpha \left(y_{k}\right)\right)}^{2}+{\left(\eta \left(y_{k}\right)\right)}^{2}\right)+\left({\left(\rho_{\xi }\left(y_{k}\right)\right)}^{2}+{\left(\rho_{\alpha }\left(y_{k}\right)\right)}^{2}+{\left(\rho_{\eta }\left(y_{k}\right)\right)}^{2}\right)\right]\\ \sum_{k=1}^{n}\left(\omega_{k}\right)\left[\left({\left(\xi \left(z_{k}\right)\right)}^{2}+{\left(\alpha \left(z_{k}\right)\right)}^{2}+{\left(\eta \left(z_{k}\right)\right)}^{2}\right)+\left({\left(\rho_{\xi }\left(z_{k}\right)\right)}^{2}+{\left(\rho_{\alpha }\left(z_{k}\right)\right)}^{2}+{\left(\rho_{\eta }\left(z_{k}\right)\right)}^{2}\right)\right] \end{array}\right\}}. \end{array}$$

**Remark 1 .**

*ω*_*k*_=1/*n* implies that ∁_*Ω*_=∁ and ∁_Ω_′=∁′.

**Theorem 3 .**

Let ∁_*Ω*_(*Y*, *Z*) be the correlation coefficient for CPFSs *Y* and *Z*. Then,

- It is symmetric, i.e., ∁_*Ω*_(*Y*, *Z*)=∁_*Ω*_(*Z*, *Y*)
- It is an FN, i.e., 0 ≤ ∁_*Ω*_(*Y*, *Z*) ≤ 1
- ∁_*Ω*_(*Y*, *Z*)=1⇔*Y*=*Z*

**Proof**

The proofs are straight forward.

**Theorem 4 .**

Let ∁_Ω_′(*Y*, *Z*) be the correlation coefficient for CPFSs *Y* and *Z*. Then,

- It is symmetric, i.e., ∁_Ω_′(*Y*, *Z*)=∁_Ω_′(*Z*, *Y*)
- It is an FN, i.e., 0 ≤ ∁_Ω_′(*Y*, *Z*) ≤ 1
- ∁_Ω_′(*Y*, *Z*)=1⇔*Y*=*Z*

**Proof**

The proofs are straight forward.

The article "An Innovative Decision-Making Approach Based on Correlation Coefficients of Complex Picture Fuzzy Sets and Their Applications in Cluster Analysis" was published in 2022. Journal: Comput Intell Neurosci.

## 4. Clustering Algorithm for Complex Picture Fuzzy Numbers

This section proposes a clustering algorithm for CPFS using newly defined concepts and formulae. In addition, the proposed clustering algorithm based on innovative structure is applied to achieve the solution for a problem involving the complex picture fuzzy information. First, some essential notions are defined.

**Definition 16 .**

A matrix ℳ=(*C*_*jk*_)_*m*×*m*_ is said to be the matrix of correlation coefficients when *Z*_*k*_ is the collection of CPFSs, and *C*_*jk*_=*C*(*Z*_*j*_, *Z*_*k*_) denotes the correlation coefficient between (*Z*_*j*_, *Z*_*k*_).

**Definition 17 .**

For a matrix of correlation coefficients ℳ, the composite matrix is symbolized as (*C*_*jk*_^*c*^)_*m*×*m*_ and defined by

(23) $$\begin{array}{c} {ℳ}^{2}=ℳ\circ ℳ={\left(C_{jk}^{c}\right)}_{m\times m}=\underset{l}{\max}\left\{\min\left(C_{jl},C_{lk}\right)\right\}. \end{array}$$

**Theorem 5 .**

Let *a*, *b* ∈ ℕ, and ℳ^*a*^, ℳ^*b*^ be matrices of correlation coefficients, then their composition matrix is also a matrix of correlation coefficients, i.e., ℳ=ℳ^*a*^∘ℳ^*b*^ is a matrix of correlation coefficients.

**Definition 18 .**

Let ℳ=(*C*_*jk*_)_*m*×*m*_ denote the matrix of correlation of coefficients, then ℳ^2^=ℳ∘ℳ⊆ℳ implies that ℳ is an equivalent matrix of correlation coefficients. The following formula defines the equivalent matrix of correlation of coefficients:

(24) $$\begin{array}{c} {ℳ}^{2}\subseteq ℳ\Rightarrow \underset{l}{\max}\left\{\min\left(C_{jl},C_{lk}\right)\right\}\leq C_{jk}. \end{array}$$

**Theorem 6 .**

For a finite natural number *a* ∈ ℕ, the recurrent *a* compositions of a matrix of correlation coefficients ℳ give an equivalent matrix of correlation coefficients ℳ^2*a*^, i.e., ℳ⟶ℳ∘ℳ=ℳ^2^⟶ℳ^2^∘ℳ^2^=ℳ^4^⟶…ℳ^*a*^∘ℳ^*a*^=ℳ^2*a*^=ℳ^2(*a*+1)^.

The equivalent matrices are similar, and they possess the same properties and information. Thus, in case of ℳ^2*a*^=ℳ^2(*a*+1)^ for some *a* ∈ ℕ, ℳ^2(*a*+1)^ preserves the structure, information, and meaning of its predecessor matrix ℳ^2*a*^. Since the equivalence matrices preserve the properties, they are calculated to categorize the attributes under consideration, which is sometimes not possible in contrary scenarios.

**Definition 19 .**

Let *α* ∈ [*a*, *b*] for any *a*, *b* ∈ [0,1]∋*a* < *b* and ℳ=(*C*_*jk*_)_*m*×*m*_ be the matrix of correlation coefficients, then an *α*-cutting matrix of ℳ is symbolized as ℳ_*α*_ and defined by

(25) $$\begin{array}{c} {ℳ}_{\alpha }={\left(\alpha C_{jk}\right)}_{m\times m}=\alpha C\left(Z_{j},Z_{k}\right)=\left\{\begin{array}{c} a\;if\;C_{jk}\leq \alpha \\ b\;if\;C_{jk}\geq \alpha \end{array}\right). \end{array}$$

Now, the clustering algorithm for CPFSs is presented and explained in a step-wise manner below.

The article "An Innovative Decision-Making Approach Based on Correlation Coefficients of Complex Picture Fuzzy Sets and Their Applications in Cluster Analysis" was published in 2022. Journal: Comput Intell Neurosci.

### 4.1. Algorithm

**Step 1 .**

For a collection of CPFSs *Z*_*k*_, construct the matrix of correlation coefficients ℳ=(*C*_*jk*_)_*m*×*m*_ by using Definition 16.

**Step 2 .**

The step targets to achieve the equivalent matrix of correlation coefficients. If ℳ holds the property, then proceed to step 3. Otherwise, the process of composition is repeated until an equivalent matrix of correlation coefficients is achieved, i.e., ℳ^2*a*^=ℳ^2(*a*+1)^, where *α* ∈ ℕ.

**Step 3 .**

Finally, the *α*-cutting matrix ℳ_*α*_ is formulated for the classification of CPFSs *Z*_*k*_. For the classification the following rules apply, “If every entry in *j*^*th*^ row and corresponding *k*^*th*^ column of *α* -cutting matrix ℳ_*α*_ are same, then the CPFSs are declared to be of the same type.”

Figure 2 portrays the process of the proposed clustering algorithm for CPFSs.

## 5. Application

In this section, an application of the proposed correlation coefficients and clustering algorithm for CPFSs is presented. The following application demonstrates an illustration of the proposed method. It can be extended and applied in several fields of science and business, where an automated and flawless decision is required. This method surpasses the uncertainties, especially in decision-making. In addition, it also automatically classifies the products/entities based on person's priorities.

### 5.1. Illustrative Example

In this illustration, we present a situation of laptop systems company who aims to categorize their computer machines by their specifications and features. Assume that the set of four laptops is denoted by *Z*={*Z*_1_, *Z*_2_, *Z*_3_, *Z*_4_}, where each *Z*_*k*_ represents a laptop, for *k*=1,2,3,4. Further, the features of interest are (i) processor, (ii) cost, (iii) battery, (iv) storage, and (v) build. Say, the set of features is *Y*={*y*_1_, *y*_2_, *y*_3_, *y*_4_, *y*_5_}, where, *y*_*k*_ represents speed, cost, battery, storage, and build for *k*=1,2,3,4 and 5, respectively. Initially, a CPFS is required for further processes. Henceforth, four different CPFSs are constructed for each laptop *Z*_*k*_ with the elements *y*_*k*_ representing the features. The complex picture fuzzy numbers are assigned to each feature by the experts and professionals according to their analysis of each product. The process of converting real-world problem into fuzzy language is called fuzzification. The process involves careful and precise analysis of the problem and its related parameters. A numerical scale for the translation of data into numeric form is constructed (see Figure 3). Each degree is assigned a number according to the scale. Since the information is being translated to complex picture fuzzy format, keeping the constraints in mind, the selection of the values for degrees is interdependent.

The article "An Innovative Decision-Making Approach Based on Correlation Coefficients of Complex Picture Fuzzy Sets and Their Applications in Cluster Analysis" was published in 2022. Journal: Comput Intell Neurosci.

Using above fuzzification process, these are the CPFSs *Z*_1_, *Z*_2_, *Z*_3_, and *Z*_4_, given in the following equations:

(26) $$\begin{array}{c} Z_{1}=\left\{\begin{array}{c} \left(y_{1},0.2e^{2\pi i\left(0.2\right)},0.3e^{2\pi i\left(0.2\right)},0.4e^{2\pi i\left(0.5\right)}\right),\left(y_{2},0.5e^{2\pi i\left(0.3\right)},0.1e^{2\pi i\left(0.2\right)},0.2e^{2\pi i\left(0.1\right)}\right),\\ \left(y_{3},0.3e^{2\pi i\left(0.2\right)},0.4e^{2\pi i\left(0.3\right)},0.2e^{2\pi i\left(0.4\right)}\right),\left(y_{4},0.5e^{2\pi i\left(0.5\right)},0.1e^{2\pi i\left(0.1\right)},0.1e^{2\pi i\left(0.1\right)}\right),\\ \left(y_{5},0.2e^{2\pi i\left(0.4\right)},0.2e^{2\pi i\left(0.1\right)},0.4e^{2\pi i\left(0.5\right)}\right) \end{array}\right\}, \end{array}$$

(27) $$\begin{array}{c} Z_{2}=\left\{\begin{array}{c} \left(y_{1},0.7e^{2\pi i\left(0.6\right)},0.2e^{2\pi i\left(0.2\right)},0.1e^{2\pi i\left(0.1\right)}\right),\left(y_{2},0.3e^{2\pi i\left(0.6\right)},0.3e^{2\pi i\left(0.3\right)},0.3e^{2\pi i\left(0.1\right)}\right),\\ \left(y_{3},0.6e^{2\pi i\left(0.6\right)},0.1e^{2\pi i\left(0.3\right)},0.2e^{2\pi i\left(0.1\right)}\right),\left(y_{4},0.7e^{2\pi i\left(0.7\right)},0.1e^{2\pi i\left(0.1\right)},0.1e^{2\pi i\left(0.1\right)}\right),\\ \left(y_{5},0.6e^{2\pi i\left(0.4\right)},0.2e^{2\pi i\left(0.2\right)},0.2e^{2\pi i\left(0.3\right)}\right) \end{array}\right\}, \end{array}$$

(28) $$\begin{array}{c} Z_{3}=\left\{\begin{array}{c} \left(y_{1},0.4e^{2\pi i\left(0.3\right)},0.2e^{2\pi i\left(0.4\right)},0.3e^{2\pi i\left(0.2\right)}\right),\left(y_{2},0.6e^{2\pi i\left(0.4\right)},0.2e^{2\pi i\left(0.3\right)},0.1e^{2\pi i\left(0.2\right)}\right),\\ \left(y_{3},0.3e^{2\pi i\left(0.4\right)},0.2e^{2\pi i\left(0.4\right)},0.4e^{2\pi i\left(0.1\right)}\right),\left(y_{4},0.6e^{2\pi i\left(0.5\right)},0.2e^{2\pi i\left(0.1\right)},0.1e^{2\pi i\left(0.1\right)}\right),\\ \left(y_{5},0.7e^{2\pi i\left(0.6\right)},0.1e^{2\pi i\left(0.1\right)},0.1e^{2\pi i\left(0.2\right)}\right) \end{array}\right\}, \end{array}$$

(29) $$\begin{array}{c} Z_{4}=\left\{\begin{array}{c} \left(y_{1},0.8e^{2\pi i\left(0.7\right)},0.1e^{2\pi i\left(0.2\right)},0.1e^{2\pi i\left(0.1\right)}\right),\left(y_{2},0.7e^{2\pi i\left(0.7\right)},0.1e^{2\pi i\left(0.2\right)},0.2e^{2\pi i\left(0.1\right)}\right),\\ \left(y_{3},0.7e^{2\pi i\left(0.8\right)},0.1e^{2\pi i\left(0.1\right)},0.1e^{2\pi i\left(0.1\right)}\right),\left(y_{4},0.2e^{2\pi i\left(0.6\right)},0.2e^{2\pi i\left(0.1\right)},0.5e^{2\pi i\left(0.3\right)}\right),\\ \left(y_{5},0.5e^{2\pi i\left(0.3\right)},0.2e^{2\pi i\left(0.3\right)},0.1e^{2\pi i\left(0.1\right)}\right) \end{array}\right\}. \end{array}$$

Further, a weighted vector for features is defined based on the priorities. A similar methodology described in Figure 3 applies for the selection of weight values of weight vector. The weight vector is *Ω*={0.3, 0.1, 0.3, 0.2, 0.1}. The weight vector plays an important role, as it describes the importance of certain properties and features. It actually depends on the priorities, which leads to a totally different outcome since the fundamental ingredients are acquired. Now, by using algorithm 4.1, the stepwise calculations are carried out. First, the matrix of the correlation coefficients is constructed, which has been calculated and presented in the following equation:

(30) $$\begin{array}{c} ℳ=\left[\begin{array}{cccc} 1 & 0.753 & 0.853 & 0.641\\ 0.753 & 1 & 0.896 & 0.917\\ 0.853 & 0.896 & 1 & 0.789\\ 0.641 & 0.916 & 0.789 & 1 \end{array}\right]. \end{array}$$

The second step focuses on acquiring the equivalence matrix of correlation coefficients. Thus, we calculate the composite matrix ℳ^2^=ℳ∘ℳ, which is given by

(31) $$\begin{array}{c} ℳ\circ ℳ=\\ {ℳ}^{2}=\left[\begin{array}{cccc} 1 & 0.853 & 0.853 & 0789\\ 0.853 & 1 & 0.896 & 0.917\\ 0.853 & 0.896 & 1 & 0.896\\ 0.789 & 0.917 & 0.896 & 1 \end{array}\right]. \end{array}$$

Since ℳ^2^ ≠ ℳ, ℳ is not an equivalence matrix of correlation coefficients. Thus, we shall find one by computing repetitive compositions of ℳ.

(32) $$\begin{array}{c} {ℳ}^{2}\circ {ℳ}^{2}={ℳ}^{4}\\ =\left[\begin{array}{cccc} 1 & 0.853 & 0.853 & 0.853\\ 0.853 & 1 & 0.896 & 0.917\\ 0.853 & 0.896 & 1 & 0.896\\ 0.853 & 0.917 & 0.896 & 1 \end{array}\right],\\ {ℳ}^{4}\circ {ℳ}^{4}={ℳ}^{8}\\ =\left[\begin{array}{cccc} 1 & 0.853 & 0.853 & 0.853\\ 0.853 & 1 & 0.896 & 0.917\\ 0.853 & 0.896 & 1 & 0.896\\ 0.853 & 0.917 & 0.896 & 1 \end{array}\right]. \end{array}$$

Hence, ℳ^4^ is an equivalence matrix, since ℳ^4^=ℳ^8^.

The article "An Innovative Decision-Making Approach Based on Correlation Coefficients of Complex Picture Fuzzy Sets and Their Applications in Cluster Analysis" was published in 2022. Journal: Comput Intell Neurosci.

In the final step, the *α*-cutting matrix ℳ_*α*_ is formulated for the classification of CPFSs *Z*_*k*_.

For *α* ∈ [0,0.853], the ℳ_*α*_ is calculated to be

(33) $$\begin{array}{c} {\left({ℳ}_{\alpha }\right)}_{1}=\left[\begin{array}{cccc} 0.853 & 0.853 & 0.853 & 0.853\\ 0.853 & 0.853 & 0.853 & 0.853\\ 0.853 & 0.853 & 0.853 & 0.853\\ 0.853 & 0.853 & 0.853 & 0.853 \end{array}\right]. \end{array}$$

For *α* ∈ [0.853, 0.896], the ℳ_*α*_ is calculated to be

(34) $$\begin{array}{c} {\left({ℳ}_{\alpha }\right)}_{2}=\left[\begin{array}{cccc} 0.896 & 0.853 & 0.853 & 0.853\\ 0.853 & 0.896 & 0.896 & 0.896\\ 0.853 & 0.896 & 0.896 & 0.896\\ 0.853 & 0.896 & 0.896 & 0.896 \end{array}\right]. \end{array}$$

For *α* ∈ [0.896, 0.917], the ℳ_*α*_ is calculated to be

(35) $$\begin{array}{c} {\left({ℳ}_{\alpha }\right)}_{3}=\left[\begin{array}{cccc} 0.917 & 0.896 & 0.896 & 0.896\\ 0.896 & 0.917 & 0.896 & 0.917\\ 0.896 & 0.896 & 0.917 & 0.896\\ 0.896 & 0.917 & 0.896 & 0.917 \end{array}\right]. \end{array}$$

For *α* ∈ [0.917, 1], the ℳ_*α*_ is calculated to be

(36) $$\begin{array}{c} {\left({ℳ}_{\alpha }\right)}_{4}=\left[\begin{array}{cccc} 1 & 0.917 & 0.917 & 0.917\\ 0.917 & 1 & 0.917 & 0.917\\ 0.917 & 0.917 & 1 & 0.917\\ 0.917 & 0.917 & 0.917 & 1 \end{array}\right]. \end{array}$$

All of the possible classifications of CPFSs *Z*_*k*_ are given in Table 1.

In clustering analysis, the classification of each entity into different types is rare. But it is clear from Table 1 that each laptop product is classified into different categories by using the proposed methods based on CPFSs. Henceforth, the efficacy of the proposed correlation of CPFSs is verified.

## 6. Experimental Comparison and Result Analysis

In the section, different experiments shall be performed to solve the above correlation coefficients problem under different frameworks such as IFSs, CIFSs, and PFSs. In order to carry out a fair comparison, the data will be taken from the previous example without any modifications. Some of the structures are limited to only membership and nonmembership functions, and others lack phase terms; therefore, some numbers will be omitted from the data.

### 6.1. Analysis of Results under IFSs and CIFSs

In this illustration, the same situation of the laptops company is presented. Since the CIFSs are the generalization of IFSs and the former is superior to the latter, the comparison will be carried out between the generalized structure and the proposed method. Instead of CPFSs, CIFSs will be used to solve the problem. The CIFSs are *Z*_1_, *Z*_2_, *Z*_3_, and *Z*_4_, given in the following equations:

(37) $$\begin{array}{c} Z_{1}=\left\{\begin{array}{c} \left(y_{1},0.2e^{2\pi i\left(0.2\right)},0.4e^{2\pi i\left(0.5\right)}\right),\left(y_{2},0.5e^{2\pi i\left(0.3\right)},0.2e^{2\pi i\left(0.1\right)}\right),\\ \left(y_{3},0.3e^{2\pi i\left(0.2\right)},0.2e^{2\pi i\left(0.4\right)}\right),\left(y_{4},0.5e^{2\pi i\left(0.5\right)},0.1e^{2\pi i\left(0.1\right)}\right),\\ \left(y_{5},0.2e^{2\pi i\left(0.4\right)},0.4e^{2\pi i\left(0.5\right)}\right) \end{array}\right\}, \end{array}$$

(38) $$\begin{array}{c} Z_{2}=\left\{\begin{array}{c} \left(y_{1},0.7e^{2\pi i\left(0.6\right)},0.1e^{2\pi i\left(0.1\right)}\right),\left(y_{2},0.3e^{2\pi i\left(0.6\right)},0.3e^{2\pi i\left(0.1\right)}\right),\\ \left(y_{3},0.6e^{2\pi i\left(0.6\right)},0.2e^{2\pi i\left(0.1\right)}\right),\left(y_{4},0.7e^{2\pi i\left(0.7\right)},0.1e^{2\pi i\left(0.1\right)}\right),\\ \left(y_{5},0.6e^{2\pi i\left(0.4\right)},0.2e^{2\pi i\left(0.3\right)}\right) \end{array}\right\}, \end{array}$$

(39) $$\begin{array}{c} Z_{3}=\left\{\begin{array}{c} \left(y_{1},0.4e^{2\pi i\left(0.3\right)},0.3e^{2\pi i\left(0.2\right)}\right),\left(y_{2},0.6e^{2\pi i\left(0.4\right)},0.1e^{2\pi i\left(0.2\right)}\right),\\ \left(y_{3},0.3e^{2\pi i\left(0.4\right)},0.4e^{2\pi i\left(0.1\right)}\right),\left(y_{4},0.6e^{2\pi i\left(0.5\right)},0.1e^{2\pi i\left(0.1\right)}\right),\\ \left(y_{5},0.7e^{2\pi i\left(0.6\right)},0.1e^{2\pi i\left(0.2\right)}\right) \end{array}\right\}, \end{array}$$

(40) $$\begin{array}{c} Z_{4}=\left\{\begin{array}{c} \left(y_{1},0.8e^{2\pi i\left(0.7\right)},0.1e^{2\pi i\left(0.1\right)}\right),\left(y_{2},0.7e^{2\pi i\left(0.7\right)},0.2e^{2\pi i\left(0.1\right)}\right),\\ \left(y_{3},0.7e^{2\pi i\left(0.8\right)},0.1e^{2\pi i\left(0.1\right)}\right),\left(y_{4},0.2e^{2\pi i\left(0.6\right)},0.5e^{2\pi i\left(0.3\right)}\right),\\ \left(y_{5},0.5e^{2\pi i\left(0.3\right)},0.1e^{2\pi i\left(0.1\right)}\right) \end{array}\right\}. \end{array}$$

The weight vector remains the same, i.e., *Ω*={0.3, 0.1, 0.3, 0.2, 0.1}. Now, the stepwise calculations are carried out by using algorithm 4.1. The matrix of the correlation coefficients is given by

(41) $$\begin{array}{c} ℳ=\left[\begin{array}{cccc} 1 & 0.751 & 0.847 & 0.655\\ 0.751 & 1 & 0.906 & 0.925\\ 0.847 & 0.906 & 1 & 0.816\\ 0.655 & 0.925 & 0.816 & 1 \end{array}\right]. \end{array}$$

Now, in the search for an equivalence matrix of correlation coefficients, compute ℳ^2^=ℳ∘ℳ.

(42) $$\begin{array}{c} ℳ\circ ℳ={ℳ}^{2}=\left[\begin{array}{cccc} 1 & 0.847 & 0.847 & 0.816\\ 0.847 & 1 & 0.906 & 0.925\\ 0.847 & 0.906 & 1 & 0.906\\ 0.816 & 0.925 & 0.906 & 1 \end{array}\right]. \end{array}$$

Since ℳ^2^ ≠ ℳ, the computation is repeated.

(43) $$\begin{array}{c} {ℳ}^{2}\circ {ℳ}^{2}={ℳ}^{4}=\left[\begin{array}{cccc} 1 & 0.847 & 0.847 & 0.847\\ 0.847 & 1 & 0.906 & 0.925\\ 0.847 & 0.906 & 1 & 0.906\\ 0.847 & 0.925 & 0.906 & 1 \end{array}\right],\\ {ℳ}^{4}\circ {ℳ}^{4}={ℳ}^{8}=\left[\begin{array}{cccc} 1 & 0.847 & 0.847 & 0.847\\ 0.847 & 1 & 0.906 & 0.925\\ 0.847 & 0.906 & 1 & 0.906\\ 0.847 & 0.925 & 0.906 & 1 \end{array}\right]. \end{array}$$

Hence, ℳ^4^ is an equivalence matrix, since ℳ^4^=ℳ^8^.

The article "An Innovative Decision-Making Approach Based on Correlation Coefficients of Complex Picture Fuzzy Sets and Their Applications in Cluster Analysis" was published in 2022. Journal: Comput Intell Neurosci.

In the final step, the *α*-cutting matrix ℳ_*α*_ is formulated for the classification of CIFSs *Z*_*k*_.

For *α* ∈ [0,0.847], ℳ_*α*_ is calculated to be

(44) $$\begin{array}{c} {\left({ℳ}_{\alpha }\right)}_{1}=\left[\begin{array}{c} \begin{array}{ccc} 0.847 & 0.847 & \begin{array}{cc} 0.847 & 0.847 \end{array}\\ 0.847 & 0.847 & \begin{array}{cc} 0.847 & 0.847 \end{array}\\ 0.847 & 0.847 & \begin{array}{cc} 0.847 & 0.847 \end{array} \end{array}\\ \begin{array}{ccc} 0.847 & 0.847 & \begin{array}{cc} 0.847 & 0.847 \end{array} \end{array} \end{array}\right]. \end{array}$$

For *α* ∈ [0.847, 0.906], ℳ_*α*_ is calculated to be

(45) $$\begin{array}{c} {\left({ℳ}_{\alpha }\right)}_{2}=\left[\begin{array}{c} \begin{array}{ccc} 0.906 & 0.847 & \begin{array}{cc} 0.847 & 0.847 \end{array}\\ 0.847 & 0.906 & \begin{array}{cc} 0.906 & 0.906 \end{array}\\ 0.847 & 0.906 & \begin{array}{cc} 0.906 & 0.906 \end{array} \end{array}\\ \begin{array}{ccc} 0.847 & 0.906 & \begin{array}{cc} 0.906 & 0.906 \end{array} \end{array} \end{array}\right]. \end{array}$$

For *α* ∈ [0.906, 0.925], ℳ_*α*_ is calculated to be

(46) $$\begin{array}{c} {\left({ℳ}_{\alpha }\right)}_{3}=\left[\begin{array}{cccc} 0.925 & 0.906 & 0.906 & 0.906\\ 0.906 & 0.925 & 0.906 & 0.925\\ 0.906 & 0.906 & 0.925 & 0.906\\ 0.906 & 0.925 & 0.906 & 0.925 \end{array}\right]. \end{array}$$

For *α* ∈ [0.925, 1], ℳ_*α*_ is calculated to be

(47) $$\begin{array}{c} {\left({ℳ}_{\alpha }\right)}_{4}=\left[\begin{array}{cccc} 1 & 0.925 & 0.925 & 0.925\\ 0.925 & 1 & 0.925 & 0.925\\ 0.925 & 0.925 & 1 & 0.925\\ 0.925 & 0.925 & 0.925 & 1 \end{array}\right]. \end{array}$$

All of the possible classifications of CIFSs *Z*_*k*_ are given in Table 2.

If we tend to solve the problem under the influence of IFSs through the methods of [25], it would lead to the following:

(48) $$\begin{array}{c} Z_{1}=\left\{\begin{array}{c} \left(y_{1},0.2,0.4\right),\left(y_{2},0.5,0.2\right),\left(y_{3},0.3,0.2\right),\left(y_{4},0.5,0.1\right),\left(y_{5},0.2,0.4\right) \end{array}\right\},\\ Z_{2}=\left\{\begin{array}{c} \left(y_{1},0.7,0.1\right),\left(y_{2},0.3,0.3\right),\left(y_{3},0.6,0.2\right),\left(y_{4},0.7,0.1\right),\left(y_{5},0.6,0.2\right) \end{array}\right\},\\ Z_{3}=\left\{\begin{array}{c} \left(y_{1},0.4,0.3\right),\left(y_{2},0.6,0.1\right),\left(y_{3},0.3,0.4\right),\left(y_{4},0.6,0.1\right),\left(y_{5},0.7,0.1\right) \end{array}\right\},\\ Z_{4}=\left\{\begin{array}{c} \left(y_{1},0.8,0.1\right),\left(y_{2},0.7,0.2\right),\left(y_{3},0.7,0.1\right),\left(y_{4},0.2,0.5\right),\left(y_{5},0.5,0.1\right) \end{array}\right\}, \end{array}$$

(49) $$\begin{array}{c} ℳ=\left[\begin{array}{cccc} 1 & 0.796 & 0.894 & 0.683\\ 0.796 & 1 & 0.883 & 0.881\\ 0.894 & 0.883 & 1 & 0.759\\ 0.683 & 0.881 & 0.759 & 1 \end{array}\right],\\ {ℳ}^{2}=\left[\begin{array}{cccc} 1 & 0.883 & 0.894 & 0.796\\ 0.883 & 1 & 0.883 & 0.881\\ 0.894 & 0.883 & 1 & 0.881\\ 0.796 & 0.881 & 0.881 & 1 \end{array}\right],\\ {ℳ}^{4}=\left[\begin{array}{cccc} 1 & 0.883 & 0.894 & 0.881\\ 0.883 & 1 & 0.883 & 0.881\\ 0.894 & 0.883 & 1 & 0.881\\ 0.881 & 0.881 & 0.881 & 1 \end{array}\right],\\ {ℳ}^{8}=\left[\begin{array}{cccc} 1 & 0.883 & 0.894 & 0.881\\ 0.883 & 1 & 0.883 & 0.881\\ 0.894 & 0.883 & 1 & 0.881\\ 0.881 & 0.881 & 0.881 & 1 \end{array}\right]. \end{array}$$

Hence, ℳ^4^ is an equivalence matrix. The classification of IFSs *Z*_*k*_ is given by

(50) $$\begin{array}{c} \alpha \in \left[0,0.881\right]\Rightarrow \left\{Z_{1},Z_{2},Z_{3},Z_{4}\right\},\\ \alpha \in \left[0.881,0.883\right]\Rightarrow \left\{Z_{1},Z_{2},Z_{3}\right\},\left\{Z_{4}\right\},\\ \alpha \in \left[0.883,0.894\right]\Rightarrow \left\{Z_{1},Z_{3}\right\},\left\{Z_{2}\right\},\left\{Z_{4}\right\},\\ \alpha \in \left[0.894,1\right]\Rightarrow \left\{Z_{1}\right\},\left\{Z_{2}\right\},\left\{Z_{3}\right\},\left\{Z_{4}\right\}. \end{array}$$

Thus, it is clear that removing the degree of abstinence and phase terms greatly affects the final results, and the classification is not as required. Although the algorithm comes to similar looking results, these processes have been carried out on incomplete information, thus leading to false outcomes.

The article "An Innovative Decision-Making Approach Based on Correlation Coefficients of Complex Picture Fuzzy Sets and Their Applications in Cluster Analysis" was published in 2022. Journal: Comput Intell Neurosci.

### 6.2. Analysis of Results under PFSs

In this experiment, the same problem is solved under the correlation coefficients of PFSs defined by Ganie et al. [30]. The PFSs are *Z*_1_, *Z*_2_, *Z*_3_, and *Z*_4_, given in Table 3.

The values of weight vector do not change; *Ω*={0.3, 0.1, 0.3, 0.2, 0.1}. By following algorithm 4.1, matrix of the correlation coefficients is found.

(51) $$\begin{array}{c} ℳ=\left[\begin{array}{cccc} 1 & 0.757 & 0.871 & 0.644\\ 0.757 & 1 & 0.882 & 0.877\\ 0.871 & 0.882 & 1 & 0.762\\ 0.644 & 0.877 & 0.762 & 1 \end{array}\right]. \end{array}$$

Now, the search for an equivalence matrix of correlation coefficients begins, and thus the matrix composition is carried out until the required matrix is obtained.

(52) $$\begin{array}{c} ℳ\circ ℳ={ℳ}^{2}=\left[\begin{array}{cccc} 1 & 0.871 & 0.871 & 0.762\\ 0.871 & 1 & 0.882 & 0.877\\ 0.871 & 0.882 & 1 & 0.877\\ 0.762 & 0.877 & 0.877 & 1 \end{array}\right]. \end{array}$$

Since, ℳ^2^ ≠ ℳ, the computation is repeated.

(53) $$\begin{array}{c} {ℳ}^{2}\circ {ℳ}^{2}={ℳ}^{4}=\left[\begin{array}{cccc} 1 & 0.871 & 0.871 & 0.871\\ 0.871 & 1 & 0.882 & 0.877\\ 0.871 & 0.882 & 1 & 0.877\\ 0.871 & 0.877 & 0.877 & 1 \end{array}\right],\\ {ℳ}^{4}\circ {ℳ}^{4}={ℳ}^{8}=\left[\begin{array}{cccc} 1 & 0.871 & 0.871 & 0.871\\ 0.871 & 1 & 0.882 & 0.877\\ 0.871 & 0.882 & 1 & 0.877\\ 0.871 & 0.877 & 0.877 & 1 \end{array}\right]. \end{array}$$

Hence, ℳ^4^ is an equivalence matrix, since ℳ^4^=ℳ^8^.

The article "An Innovative Decision-Making Approach Based on Correlation Coefficients of Complex Picture Fuzzy Sets and Their Applications in Cluster Analysis" was published in 2022. Journal: Comput Intell Neurosci.

Finally, the *α*-cutting matrix ℳ_*α*_ is formulated for the classification of PFSs *Z*_*k*_.

For *α* ∈ [0,0.871], ℳ_*α*_ is calculated to be

(54) $$\begin{array}{c} {\left({ℳ}_{\alpha }\right)}_{1}=\left[\begin{array}{c} \begin{array}{ccc} 0.871 & 0.871 & \begin{array}{cc} 0.871 & 0.871 \end{array}\\ 0.871 & 0.871 & \begin{array}{cc} 0.871 & 0.871 \end{array}\\ 0.871 & 0.871 & \begin{array}{cc} 0.871 & 0.871 \end{array} \end{array}\\ \begin{array}{ccc} 0.871 & 0.871 & \begin{array}{cc} 0.871 & 0.871 \end{array} \end{array} \end{array}\right]. \end{array}$$

For *α* ∈ [0.871, 0.877], ℳ_*α*_ is calculated to be

(55) $$\begin{array}{c} {\left({ℳ}_{\alpha }\right)}_{2}=\left[\begin{array}{c} \begin{array}{ccc} 0.877 & 0.871 & \begin{array}{cc} 0.871 & 0.871 \end{array}\\ 0.871 & 0.877 & \begin{array}{cc} 0.877 & 0.877 \end{array}\\ 0.871 & 0.877 & \begin{array}{cc} 0.877 & 0.877 \end{array} \end{array}\\ \begin{array}{ccc} 0.871 & 0.877 & \begin{array}{cc} 0.877 & 0.877 \end{array} \end{array} \end{array}\right]. \end{array}$$

For *α* ∈ [0.877, 0.882], ℳ_*α*_ is calculated to be

(56) $$\begin{array}{c} {\left({ℳ}_{\alpha }\right)}_{3}=\left[\begin{array}{cccc} 0.882 & 0.877 & 0.877 & 0.877\\ 0.877 & 0.882 & 0.882 & 0.877\\ 0.877 & 0.882 & 0.882 & 0.877\\ 0.877 & 0.877 & 0.877 & 0.882 \end{array}\right]. \end{array}$$

For *α* ∈ [0.882, 1], ℳ_*α*_ is calculated to be

(57) $$\begin{array}{c} {\left({ℳ}_{\alpha }\right)}_{4}=\left[\begin{array}{cccc} 1 & 0.882 & 0.882 & 0.882\\ 0.882 & 1 & 0.882 & 0.882\\ 0.882 & 0.882 & 1 & 0.882\\ 0.882 & 0.882 & 0.882 & 1 \end{array}\right]. \end{array}$$

All of the possible classifications of PFSs *Z*_*k*_ are given in Table 4.

In the light of the above experimental results, it is observed that the CIFS-based correlation coefficient technique classified the products into the same categories as the proposed method. However, their numerical scores are different from those in the proposed work. An important conclusion is that (i) the designation of three functions (membership, abstinence, and nonmembership) to the entities affects the results. (ii) The similar categorization implies that the proposed structure is the generalization of CIFSs. Hence, it will always provide more accurate and reliable results due to its greater structure.

In the case of the correlation coefficient based on PFS, the phase terms are completely neglected. The final outcomes are different from the ones achieved by using the proposed method. Besides different output values and class values, the categories are also not the same. The final remarks are stated as: (i) the phase terms drastically affect the final outcomes. (ii) The proposed method is far superior to the PFS-based method due to its complex structure. (iii) The results of the proposed method are more reliable because it takes time into consideration.

The article "An Innovative Decision-Making Approach Based on Correlation Coefficients of Complex Picture Fuzzy Sets and Their Applications in Cluster Analysis" was published in 2022. Journal: Comput Intell Neurosci.

It is perceived that the proposed correlation coefficient for CPFS is a complete package. It takes all sorts of information into account and thus yields a relatively perfect and reliable outcome, whereas the other methods fail to comply with the required levels of accuracy. Even though the results look similar, their reliability differs. As correlation coefficient algorithms for PFSs [30] lack the phase terms, CIFSs lack the abstinence degrees, and IFSs [25] fall short due to nonapplicability to problems involving abstinence degrees and phase terms. Thus, their results do not meet the mandatory altitudes due to the loss of information in those methods. A thorough comparison of the final results is presented in Table 5.

### 6.3. Comparative remarks

In the following sections, the limitations of the methods based on present structures are given along with the advantages of the proposed methods.

#### 6.3.1. Limitations of Present Structures

- The fuzzy set (FS) and complex FS (CFS) only describe the membership of an entity and miss out all the other details. This deficiency limits their abilities to model many real-life scenarios.
- Even with membership and nonmembership functions, the IFSs and CIFSs cannot model all sorts of circumstances because there is no representative for abstinent remarks. These limitations make them unusable in certain situations.
- The absence of the abstinence function in PFSs also bounds their propensity to solve problems that take time into consideration.
- The deficits in the present structures, such as FS, CFS, IFS, CIFS, and PFS, make their correlation coefficients inoperable in particular settings.

#### 6.3.2. Advantages of Proposed Structure

- Speaking of structure, the proposed CPFSs are superior to all of the existing notions because they model three different functions that are membership, abstinence, and nonmembership. In addition, their complex-valued structure gives them an edge on simple-valued frameworks. In total, they have six functions, which is the greatest for any structure in the theory of FSs.
- The CPFSs are the generalization of FSs, CFSs, IFSs, CIFSs, and PFSs. In CPFSs, putting certain functions equal to zero will still solve the given problem in the aforementioned environments.
- The correlation coefficients proposed in this paper for CPFSs are also generalizations of the correlation coefficients for IFS, CIFS, and PFS. Thus, the proposed methods have the ability to solve the problems in other frameworks.

The article "An Innovative Decision-Making Approach Based on Correlation Coefficients of Complex Picture Fuzzy Sets and Their Applications in Cluster Analysis" was published in 2022. Journal: Comput Intell Neurosci.

## 7. Conclusions

In this research article, some basic notions of fuzzy set theory were defined. Moreover, some novel ideas were established that include information energy of a complex picture fuzzy set (CPFS), correlation among CPFSs, correlation coefficients of CPFSs, matrices of correlation coefficients, composition matrices of correlation coefficients, and equivalent matrices. Further, a clustering algorithm was first proposed for complex structures, i.e., complex picture fuzzy information, which can also deal with all sorts of fuzzy information such as fuzzy, complex fuzzy, intuitionistic fuzzy, complex intuitionistic fuzzy, and picture fuzzy information. The major benefit of the proposed framework is that it can model up to three aspects of an entity with respect to some variable. Furthermore, it can process real-valued data as well as complex-valued data as compared to the preexisting methods that only deal with real-valued data and lack the phase terms. Additionally, this article proposed an application of the proposed concepts and clustering algorithm that exemplified the way of classifying similar items on the basis of features. In the end, different experiments were carried out to solve the clustering problem by using other existing techniques. As a result, the proposed method stood out, and its work was validated through a deep analysis of experimental results. The proposed technique and structures can be used for all types of data and applied to pattern recognition in buildings' construction, categorizing and analyzing the types of masks based on material, and many others. Aiming at the expansion of the range of applications, these concepts will be extended in the future by making amendments to the structures.

## Figures and Tables

**Figure 1:** CPFSs and their generalizations.

**Figure 2:** Flowchart for the proposed clustering algorithm.

**Figure 3:** A numerical scale for fuzzification.

**Table 1:** The classification of four sets of laptops on the basis of proposed correlation coefficients.

*α*	Classification
*α* ∈ [0,0.853]	{*Z*_1_, *Z*_2_, *Z*_3_, *Z*_4_}
*α* ∈ [0.853, 0.896]	{*Z*_1_}, {*Z*_2_, *Z*_3_, *Z*_4_}
*α* ∈ [0.896, 0.917]	{*Z*_1_}, {*Z*_3_}, {*Z*_2_, *Z*_4_}
*α* ∈ [0.917, 1]	{*Z*_1_}, {*Z*_2_}, {*Z*_3_}, {*Z*_4_}

**Table 2:** The classification of four sets of laptops on the basis of correlation coefficients under complex intuitionistic fuzzy information.

*α*	Classification
*α* ∈ [0,0.847]	{*Z*_1_, *Z*_2_, *Z*_3_, *Z*_4_}
*α* ∈ [0.847, 0.906]	{*Z*_1_}, {*Z*_2_, *Z*_3_, *Z*_4_}
*α* ∈ [0.906, 0.925]	{*Z*_1_}, {*Z*_3_}, {*Z*_2_, *Z*_4_}
*α* ∈ [0.925, 1]	{*Z*_1_}, {*Z*_2_}, {*Z*_3_}, {*Z*_4_}

The article "An Innovative Decision-Making Approach Based on Correlation Coefficients of Complex Picture Fuzzy Sets and Their Applications in Cluster Analysis" was published in 2022. Journal: Comput Intell Neurosci.

**Table 3:** Features of laptops in terms of PFS.

	**y**_1_	**y**_2_	**y**_3_	**y**_4_	**y**_5_
*Z*_1_	(0.2, 0.3, 0.4)	(0.5, 0.1, 0.2)	(0.3, 0.4, 0.2)	(0.5, 0.1, 0.1)	(0.2, 0.2, 0.4)
*Z*_2_	(0.7, 0.2, 0.1)	(0.3, 0.3, 0.3)	(0.6, 0.1, 0.2)	(0.7, 0.1, 0.1)	(0.6, 0.2, 0.2)
*Z*_3_	(0.4, 0.2, 0.3)	(0.6, 0.2, 0.1)	(0.3, 0.2, 0.4)	(0.6, 0.2, 0.1)	(0.7, 0.1, 0.1)
*Z*_4_	(0.8, 0.1, 0.1)	(0.7, 0.1, 0.2)	(0.7, 0.1, 0.1)	(0.2, 0.2, 0.5)	(0.5, 0.2, 0.1)

**Table 4:** The classification of four sets of laptops on the basis of correlation coefficients under picture fuzzy information.

*α*	Classification
*α* ∈ [0,0.847]	{*Z*_1_, *Z*_2_, *Z*_3_, *Z*_4_}
*α* ∈ [0.847, 0.906]	{*Z*_1_}, {*Z*_2_, *Z*_3_, *Z*_4_}
*α* ∈ [0.906, 0.925]	{*Z*_1_}, {*Z*_2_, *Z*_3_}, {*Z*_4_}
*α* ∈ [0.925, 1]	{*Z*_1_}, {*Z*_2_}, {*Z*_3_}, {*Z*_4_}

**Table 5:** A complete comparison for the outcomes through different approaches.

Proposed approach		Approach of [30] using PFS	
*α*	Classification	*α*	Classification

[0,0.853]	{*Z*_1_, *Z*_2_, *Z*_3_, *Z*_4_}	[0,0.847]	{*Z*_1_, *Z*_2_, *Z*_3_, *Z*_4_}
[0.853, 0.896]	{*Z*_1_}, {*Z*_2_, *Z*_3_, *Z*_4_}	[0.847, 0.906]	{*Z*_1_}, {*Z*_2_, *Z*_3_, *Z*_4_}
[0.896, 0.917]	{*Z*_1_}, {*Z*_3_}, {*Z*_2_, *Z*_4_}	[0.906, 0.925]	{*Z*_1_}, {*Z*_2_, *Z*_3_}, {*Z*_4_}
[0.917, 1]	{*Z*_1_}, {*Z*_2_}, {*Z*_3_}, {*Z*_4_}	[0.925, 1]	{*Z*_1_}, {*Z*_2_}, {*Z*_3_}, {*Z*_4_}

CIFS		Approach of [25] using IFS	
*α*	Classification	*α*	Classification

[0,0.847]	{*Z*_1_, *Z*_2_, *Z*_3_, *Z*_4_}	[0,0.881]	{*Z*_1_, *Z*_2_, *Z*_3_, *Z*_4_}
[0.847, 0.906]	{*Z*_1_}, {*Z*_2_, *Z*_3_, *Z*_4_}	[0.881, 0.883]	{*Z*_1_, *Z*_2_, *Z*_3_}, {*Z*_4_}
[0.906, 0.925]	{*Z*_1_}, {*Z*_3_}, {*Z*_2_, *Z*_4_}	[0.883, 0.894]	{*Z*_1_, *Z*_3_}, {*Z*_2_}, {*Z*_4_}
[0.925, 1]	{*Z*_1_}, {*Z*_2_}, {*Z*_3_}, {*Z*_4_}	[0.894, 1]	{*Z*_1_}, {*Z*_2_}, {*Z*_3_}, {*Z*_4_}

## Data Availability

No data were used to support this study.
